The article "PAK5 facilitates the proliferation, invasion and migration in colorectal cancer cells" was retracted in 2024. Reasons: duplicated images; duplicated data; overlap with earlier publications; original data or images not available.

# PAK5 facilitates the proliferation, invasion and migration in colorectal cancer cells

**DOI:** 10.1002/cam4.3084

**Published:** 2020-05-08

**Authors:** Silin Huang, Ying Zhu, Chunfei Wang, Xiaxi Li, Xiaobing Cui, Sufang Tu, Lijuan You, JingWen Fu, Zemin Chen, Wei Hu, Wei Gong

**Affiliations:** ^1^ Department of Gastroenterology Shenzhen Hospital Southern Medical University Shenzhen Guangdong China; ^2^ Endoscopy Center The Seventh Affiliated Hospital of Sun Yat‐Sen University Shenzhen Guangdong China; ^3^ Department of Anaesthesia and Intensive Care The Chinese University of Hong Kong Hong Kong

**Keywords:** colorectal cancer, invasion, migration, PAK5, proliferation

## Abstract

Colorectal cancer (CRC) is the third‐most common cancer around the world, accounting for approximately 10% of cancer‐related mortality. Deeper molecular understanding of colorectal carcinogenesis will provide evidences for identification of early diagnostic indicators and novel therapeutic strategies for CRC treatment. The p21^cdc42/rac1^‐activated kinase 5 (PAK5) has been reported to be involved in a variety of tumor‐promoting behaviors, whereas the underlying mechanisms of PAK5 in CRC progression are still obscure. Our current study revealed an upregulated expression of PAK5 in human CRC tissues as compared with normal adjacent biopsies, which was associated with tumor progression and metastasis. We further unraveled that inhibition of PAK5 was correlated with restrained proliferation, migration, and invasion of CRC cells in vitro and in vivo. Moreover, we showed an indispensable role of PAK5 in interacting with Cdc42 and Integrin β1, β3, thus, to facilitate the migration and invasion of CRC cells. Collectively, we pointed out a potential of PAK5 to serve as a novel therapeutic target in restricting CRC proliferation and metastasis. The uncovered mechanisms will deepen the comprehension with regard to the mechanisms of CRC progression, as well as providing new insights for therapeutic intervention in colorectal cancer.

## Graphical abstract

PAK5 was highly expressed in human CRC samples, which was correlated with cancer progression and metastasis. Inhibition of PAK5 was associated with restrained tumor cell proliferation, migration, and invasion in vitro and in vivo models. Interacting with Cdc42 and integrin β1 and β3 was indispensable for PAK5 to facilitate the migration and invasion of CRC cells.

## 1 INTRODUCTION

Colorectal cancer (CRC) is currently the third‐most predominant malignancy and the fourth leading cause of cancer‐related mortality, accounting for approximately 1 000 000 new cases and over 394 000 deaths worldwide annually.^1^, ^2^ Poor life habits such as smoking, low physical activities, and excessive consumption of red meat may attribute to the increased incidence of CRC in the past decades.^3^, ^4^ Currently, laparoscopic surgery for primary CRC and resection combined with chemoradiotherapy for metastatic CRC are still the mainstay curative treatment for patients.^5^ Nevertheless, there is little alteration in terms of cure rates and long‐term survival regardless of the great advancement in surgical and medical therapies in the last couple of years.^6^ Early diagnosis has a profound effect on CRC‐related mortality. The 5‐year survival rate for early CRC patients is around 90%, whereas it decreases to less than 14% in patients diagnosed with advanced distant metastases.^7^ Deeper molecular understanding of colorectal carcinogenesis offers novel perspective for identification of early diagnostic indicators and therapeutic strategies for CRC treatment,^8^ with a great potential to improve the outcome and prognosis of such disease. However, details of pathogenesis in CRC still largely remain obscure.

p21^cdc42/rac1^‐activated kinases (PAKs), a binding protein of small GTPases, were firstly identified as a brain‐specific kinase. Soon, they are emerged as oncogenic mediators involving a variety of signaling routes, which are required for tumorigenesis.^9^ Upon overexpression, or persistent activation by the upstream regulators, including the cell division control protein 42 (Cdc42) and Rho family GTPases RAC, PAK isoforms participate in multiple tumorigenic cascades, leading to a series of tumor‐promoting behaviors, including stimulation of cell proliferation, apoptosis evasion, and facilitating invasion and metastasis.^9^, ^10^ Based on the sequences and structural discrepancies, six PAK family members can be subdivided into two groups, group Ⅰ (PAK1‐3) and group Ⅱ (PAK4‐6).^11^ All PAK members are featured as an N‐terminal Cdc42/Ras interactive binding (CRIB) domain and a well‐conserved C‐terminal catalytic domain harboring a single phosphorylation site,^12^ although group Ⅰ and group Ⅱ are activated via distinct manners.

The article "PAK5 facilitates the proliferation, invasion and migration in colorectal cancer cells" was retracted in 2024. Reasons: duplicated images; duplicated data; overlap with earlier publications; original data or images not available.

PAK5 (also known as PAK7), located in the *Homo sapiens* 20p12 chromosomal locus and encodes a 80 kDa protein, was initially characterized as a brain‐specific kinase, which contributes to filopodia formation in nerve cells.^13^, ^14^ As the last identified and the least understood PAK family member, PAK5 mainly distributes on mitochondria and nucleus.^15^ Despite its original identification in brain neuronal cells, accumulating evidences pointed out a deep involvement of PAK5 in tumorigenesis, including the modulation of cytoskeleton alteration, antiapoptosis, and promoting cell growth in a variety of tumor cells such as pancreatic and hepatic cancers.^16^, ^17^ Several PAK family members have been proved to be involved in CRC progression. It was showed that PAK1 expression drives the development of colorectal adenoma to carcinoma.^18^ By contrast, kinase‐inactivated PAK4 prevents oncogenic Ras‐induced transformation, resulting in growth inhibition of HCT116 cells.^19^ We are among the first to elucidate an aberrant expression of PAK5 in CRC, which is closely related to its malignant progression.^20^ Moreover, we showed that endogenous expression of PAK5 attenuated camptothecin‐induced apoptosis through inhibition of Caspase‐8 activity in CRC cells.^21^ However, the underlying mechanisms of PAK5 in CRC progression still remain to be fully elucidated.

In this study, PAK5 expression in various CRC cell lines and patients’ specimens (colorectal cancer tissues vs paired noncancerous tissues) were evaluated. Our data unraveled a relatively high expression level of PAK5 in CRC tissues as compared with normal adjacent biopsies, which was correlated with cancer progression and metastasis. Inhibition of PAK5 led to restrained tumor cell growth, migration, and invasion. Moreover, our data revealed that interacting with Cdc42 and Integrin β1, β3 was indispensable for PAK5 to facilitate the migration and invasion of CRC cells. These uncovered mechanisms will further our understanding with regard to the involvement of PAK5 in CRC progression, which may provide therapeutic implications in CRC treatment.

## 2 MATERIALS AND METHODS

### 2.1 Cell culture and clinical specimens

SW480, LS174T, RKO, LOVO cells (DMEM, 10% FBS), HT29, NCM460 (McCoy's 5A, 10% FBS), HCT116, and DLD1 (RPMI‐1640, 10% FBS) were purchased from ATCC and maintained at 37℃ with 5% CO_2_.

All clinical samples utilized in this study, including primary CRC tissues and paired‐adjacent noncancerous colon tissues further than 5 cm, were collected from patients undergoing radical colon resection at the Department of Gastroenterology, Shenzhen Hospital, Southern Medical University (Guangdong, China). Fresh samples were frozen in liquid nitrogen immediately after resection and stored at −80℃. Samples were histologically stained with hematoxylin and eosin, and evaluated by experienced gastrointestinal pathologists for histological grade of cancers based on criteria set by the World Health Organization. Normal colorectal mucosa was defined as all straight, nonbranching crypts with histopathologically normal cells. All protocols were approved by the Ethic Committee of Southern Medical University (NYSZYYEC20190013) after obtaining patients’ informed consent. Samples details were summarized in Table S1.

The article "PAK5 facilitates the proliferation, invasion and migration in colorectal cancer cells" was retracted in 2024. Reasons: duplicated images; duplicated data; overlap with earlier publications; original data or images not available.

### 2.2 Plasmids construction and transfection

The following two PCR primers were designed to clone the full‐length PAK5 from a human placenta cDNA library: forward primer 5′‐CCG AAT TCA TGT TTG GGA AGA AAA AGA A‐3′ with addition of EcoRI restriction enzyme site; and the reverse primer: 5′‐ATC TAG AGT CAC GAG GCT CTC TGA TAC TCC‐3′ with addition of XbaI site. Full‐length PAK5 was cloned into the EcoRI‐XbaI sites of mammalian expression vector pCDNA3.0 (Thermo). PAK5 (K478M) was generated by site‐directed mutagenesis and contains a lysine‐to‐methionine substitution at amino acid 478 (Stratagene QuickChange Kit). PAK5△CRIB, corresponding to amino acids 9 to 53, lacking the CRIB domain and PAK5△IBD, corresponding to amino acids 634 to 658, lacking the Integrin‐binding domain (IBD) were both generated by PCR with PAK5 cDNA as the template. For plasmids transfection, cells seeded in 6‐well plates with 60%‐70% confluence were transfected by jetPRIME (Polyplus transfection) according to the standard protocols.

### 2.3 RNA isolation and reverse transcription, quantitative real‐time PCR (qRT‐PCR)

Total RNA was harvested and extracted with Trizol Reagent (Thermo) according to the manufacturers’ instruction. mRNA reverse transcription was performed using the PrimeScript RT Master Mix (Takara). mRNA levels were determined by SYBR Green Ⅱ (Takara) with a 7500 Real‐time PCR system (Life technologies). Relative quantitation of PAK5 was normalized to β‐Actin levels. The primer sequences were as follows: PAK5 forward, 5′‐TAT CTG GCC CGT CCA ACT TTG‐3′; PAK5 reverse, 5′‐GGG AAG GCC GGT AAA CTT CTG‐3′; β‐Actin forward, 5′‐CAT GTA CGT TGC TAT CCA GGC‐3′; and β‐Actin reverse, 5′‐CTC CTT AAT GTC ACG CAC GAT‐3′. All reactions were run in triplicate. The relative gene expression was calculated using the comparative threshold cycle (*C*_T_) method (Gene fold change = 2^−△△^ *^C^*_T_, △△*C*_T_ = [(*C*_T_ gene of interest—*C*_T_ internal control) sample A—(*C*_T_ gene of interest—*C*_T_ internal control) sample B]).

### 2.4 Cell proliferation assay

The Cell Counting Kit 8 (CCK‐8) was utilized to measure cell viability. Briefly, cells were prepared in a 96‐well plate (100 μL/well) and cultured in 37℃ with 5% CO_2_ after transfection. Ten μL of CCK‐8 solution was added to each well, and cells were incubated for 2 hours. Absorbance were then measured at 460 nm to calculate the cell viability. Experiments were repeated for three times.

### 2.5 Colony formation assay

A total of 1000 cells were plated per well in 6‐well plates and cultured for 1 week after transfection. Medium was removed. Cells were rinsed with PBS. Following fixation, 0.5% crystal violet solution was added, and incubated at room temperature (RT) for 2 hours. Colony numbers were calculated. Experiments were repeated for three times.

The article "PAK5 facilitates the proliferation, invasion and migration in colorectal cancer cells" was retracted in 2024. Reasons: duplicated images; duplicated data; overlap with earlier publications; original data or images not available.

### 2.6 Transwell cell migration and invasion assays

Two‐chamber plates with 8 μm pore size insert were modified for cell migration and invasion assays. Inserts coated with or without Matrigel were applied for migration or invasion assays, respectively. After transfection, cells were incubated in the transwell plates for 15 hours (Migration assay) or 24 hours (Invasion assay), then fixed by 5% glutaraldehyde for 10 minutes, and stained by 1% crystal violet in 2% ethanol for 20 minutes. The number of cells penetrating through the pores was recorded under a microscope and analyzed using ImageJ software. Experiments were repeated for three times.

### 2.7 Wound healing assay

Cells seeded in 6‐well plate were grown in complete medium for 24 hours to reach 90% confluence as a monolayer. A sterile 200 μL pipette tip was used to gently and slowly scratch the monolayer across the center of well. Photos were taken for the wound using a microscope at indicated time points. Assays were performed three times.

### 2.8 Xenograft mouse metastatic model

The BALB/c female nude mice purchased from Beijing Huafukang Bioscience (Beijing, China) were randomly arranged into four groups (n = 5 per group). Stable HCT116 cells (pLKO.1_*Ctrl* and pLKO.1_*shPAK5*) and SW480 cells (pLenti_*mock* and pLenti_*PAK5*) were concentrated to 3 × 10^6^/100 μL PBS and administrated orthotopically to mice cecum. Tumor volumes were assessed and recorded every 5 days. All mice were sacrificed. Livers were excised and photographed after 25 days. The number of metastatic tumors per liver was counted. Tumor samples were then treated for immunohistochemical or immunofluorescent staining.

### 2.9 Western blotting and immunoprecipitation

We performed western blotting assay as previously described.^22^, ^23^ Briefly, tissues or cells were washed with precool PBS, then lysed in lysis buffer containing proteasome and phosphatase inhibitors for 30 minutes. Cell lysate was collected after centrifuging at 13 000 rpm at 4°C for 30 minutes to remove the debris, then transferred to a fresh tube. Protein concentrations were normalized using a Bio‐rad protein assay kit. Twenty μg protein samples was boiled and loaded on a SDS‐PAGE following a standard protocol. Gels were transferred into PVDF membranes. 5% Non‐fat milk for 1 hour at RT was applied to block the nonspecific binding. PVDF membranes were incubated overnight at 4°C with indicated antibodies, following incubated with the diluted HRP‐conjugated secondary antibody for 1 hour at RT. PVDF membranes were incubated with ECL, then exposed to the X‐ray film to detect the targeted proteins. The immunoprecipitation assays were carried out following the standard instruction: in brief, 5 μg antibody diluted in antibody binding and washing buffer was incubated with Dynabeads™ magnetic beads. 200 μg cell lysates containing the antigen were added to the magnetic bead‐antibody complex and incubated overnight at 4℃. Beads were collected and resuspended in elution buffer. Proteins were eluted by boiling in SDS sample buffer and subjected to western blotting, then probed with specific antibodies.

The article "PAK5 facilitates the proliferation, invasion and migration in colorectal cancer cells" was retracted in 2024. Reasons: duplicated images; duplicated data; overlap with earlier publications; original data or images not available.

### 2.10 Statistical analysis

All data presented as the mean ± SD Differences between two groups were compared by the Student's *t* test. Paired t test was employed to analyze the mRNA expression levels of PAK5 between CRC and adjacent noncancerous samples. Multiple‐group comparisons were made by the one‐way analysis of variance (ANOVA) followed by the Tukey's *t* test. Statistical significance was considered as *P* values were less than .05.

## 3 RESULTS

### 3.1 Upregulated expression of PAK5 in human colorectal cancer

The expression levels of PAK5 in primary CRC tissues and colorectal cancer cells were firstly determined. PAK5 mRNA expression was evaluated in 43 cases of primary CRC tissues paralleled with adjacent noncancerous specimens by qRT‐PCR, showing a significantly upregulated expression in tumor samples (72.1%) vs normal adjacent tissues (Figure 1A). Western blotting results further confirmed the upregulation of PAK5 at protein level in primary CRCs as compared with normal adjacent samples (Figure 1B). Consistently, immunohistochemistry (IHC) analysis also showed that, in contrast to low expression of PAK5 in normal colon mucosa and adjacent noncancerous tissues, we detected a significantly upregulated PAK5 level in CRC specimens (Figure 1C). Moreover, in vitro experiments revealed that, distinct from normal human colon epithelial cell line (NCM460), significantly increased PAK5 expression levels were detected in all seven colorectal cancer cells, including SW480, HT29, LS174T, RKO, HCT116, LOVO, and DLD1 (Figure 1D). Next, we analyzed the levels of PAK5 at different tumor/node/metastasis (TNM) stages and discovered that PAK5 expression in stage Ⅲ/Ⅳ was much higher than those in stage Ⅰ/Ⅱ, suggesting a correlation of PAK5 with CRC tumor progression (Figure 1E).

**Figure 1:** PAK5 expression was upregulated in human CRC cancer. A, qRT‐PCR analysis of PAK5 mRNA levels in 43 primary CRC samples normalized by the adjacent normal tissues. B, PAK5 protein levels were determined by western blots in 8 CRC samples and normal adjacent tissues. α‐Tubulin acts as the internal control. C, Representative IHC staining of PAK5 in normal and CRC tumor tissues was shown. Scale bars represent 100 μm. D, PAK5 protein levels were determined by western blots in 7 CRC cell lines and 1 normal human colon epithelial cell line. E, Relative PAK5 mRNA levels in 43 CRC samples with early TNM stages (Ⅰ/Ⅱ) and advanced stages (Ⅲ/Ⅳ). The quantitative data were presented as means ± SD from three independent experiments. ^*^ *P* < .05; ^**^ *P* < .01; ^***^ *P* < .001

The article "PAK5 facilitates the proliferation, invasion and migration in colorectal cancer cells" was retracted in 2024. Reasons: duplicated images; duplicated data; overlap with earlier publications; original data or images not available.

### 3.2 PAK5 facilitated proliferation, migration, and invasion in CRC cells

To assess the oncogenic potential of PAK5 in CRC, we employed siRNA to selectively reduce its protein expression in HCT116 and RKO cells (Figure 2A,D). Knockdown of PAK5 remarkably prevented cell viability (Figure 2B,E) and clonogenicity (Figure 2C,F). Moreover, annexin V/7‐AAD staining assay showed that ectopic expression of PAK5 enabled SW480 and HT‐29 cells to be resistant to 5‐fluorouracil (5‐FU)‐induced apoptosis (Figure 2G,H), indicating that PAK5 potentiated CRC cells proliferation and survival capability.

**Figure 2:** PAK5 promoted proliferation and attenuated 5‐FU‐induced apoptosis in CRC cells. A, D, PAK5 protein levels in transiently transfected HCT116 and RKO cells were evaluated by western blots. B, E, HCT116 and RKO cell proliferation were determined by CCK‐8 assays after transfection with negative control or PAK5 siRNA. Absorbances were recorded every day for 7 d. C, F, Colony formation ability of HCT116 and RKO cells was assessed after transient transfection with negative control or PAK5 siRNA for 7 d. Colony number for each group was counted and analyzed. G, H, The ratio of apoptotic cell death was measured and quantified by Annexin V/7‐AAD staining assay in 5‐FU‐treated SW480 and HT‐29 cells after transient transfection with empty vector or PAK5 plasmid. The quantitative data were presented as means ± SD from three independent experiments. ^**^ *P* < .01; ^***^ *P* < .001

The effect of PAK5 on CRC cell motility was then assessed. Cell migration and invasion were measured using transwell assay. We observed weakened migration and invasion abilities in HCT116 cells after silenced with PAK5 (Figure 3A). On the contrary, PAK5 overexpression significantly enhanced SW480 cell capability of penetrating through the inserts (Figure 3C,D). Consistently, the wound‐healing assays revealed that knockdown of PAK5 markedly prevented HCT116 cell migration (Figure 3B), whereas ectopic PAK5 expression in SW480 cells showed the opposite effects (Figure 3E). Next, statistical analysis study uncovered that high PAK5 level was associated with CRC metastasis (Figure 3F). Overall, our data demonstrated a facilitating effect of PAK5 in CRC cell migration and invasion.

The article "PAK5 facilitates the proliferation, invasion and migration in colorectal cancer cells" was retracted in 2024. Reasons: duplicated images; duplicated data; overlap with earlier publications; original data or images not available.

**Figure 3:** PAK5 facilitated the migration and invasion of CRC cells. A, HCT116 cells migration and invasion after transient transfection with negative control or PAK5 siRNA were detected by transwell assays. Scale bars represent 100 μm. B, Representative images of HCT116 cells wound healing distance of shift after transient transfection with negative control or PAK5 siRNA were showed. Scale bars represent 100 μm. C, PAK5 protein levels in transiently transfected SW480 cells were detected by western blots. GAPDH acts as the internal control. D, SW480 cells migration and invasion after transient transfection with empty vector or PAK5 plasmid were detected by transwell assays. Scale bars represent 100 μm. E, Representative images of SW480 cells wound healing distance of shift after transient transfection with empty vector or PAK5 plasmid were showed. Scale bars represent 100 μm. F, Relative PAK5 mRNA expression in 43 CRC samples with metastatic and nonmetastatic tumor status. The quantitative data were presented as means ± *SD* from three independent experiments. ^*^ *P* < .05; ^**^ *P* < .01

### 3.3 PAK5 directly interacted with Cdc42 and Integrin β1, β3

The Rho family GTPases Cdc42 and cell surface glycoprotein Integrins are established to be related to cell mobility.^24^, ^25^, ^26^ Microinjection of activated Cdc42 into Swiss 3T3 fibroblasts has been reported to induce the formation of filopodia,^27^ while Integrins exhibit a marked impact on cell migration and adhesion through binding with Integrins ligands to transmit signals into the cells, resulting in cytoskeletal reorganization and gene expression.^28^ PAK family members such as PAK1 and PAK4 have been shown to be involved in cytoskeletal regulation by interacting with Cdc42 or Integrins.^29^, ^30^ Benjamin et al ever reported an indispensable role of PAK in the Integrin signaling transmission in *Drosophila*.^31^ Similarly, PAK1 has been identified to interact with Integrin β1 to promote cell migration, which was negatively modulated by Nischarin, a binding partner of Integrins.^32^ In this study, we performed the coimmunoprecipitation (co‐IP) assays, trying to determine whether PAK5 can directly interact with Cdc42 and Integrin β1, β3 in CRC cells. As shown in Figure 4A,C, PAK5 as the bait protein efficiently coprecipitated with Cdc42 and Integrin β1, β3 in HCT116 cells. By contrast, PAK5 could also be captured by Cdc42 (Figure 4B) and Integrin β1, β3 (Figure 4D,E). Moreover, confocal microscope imaging confirmed that PAK5 colocalized with Cdc42 (Figure 4F) and Integrin β1, β3 (Figure 4G) in the lamellipodial focal adhesions in HCT116 cells. Thus, our results substantiated a vital role of PAK5 in cell motility in HCT116 cells.

The article "PAK5 facilitates the proliferation, invasion and migration in colorectal cancer cells" was retracted in 2024. Reasons: duplicated images; duplicated data; overlap with earlier publications; original data or images not available.

**Figure 4:** PAK5 directly interacted with Cdc42 and Integrin β1, β3. A‐B The interaction between PAK5 and CDC42 was detected by co‐IP assays in HCT116 cells. C‐E, The interaction between PAK5 and Integrin β1, β3 was detected by co‐IP assays in HCT116 cells. F‐G, Representative immunofluorescence images of PAK5 colocalized with Cdc42 and Integrin β1, β3 in HCT116 cells were presented. Arrows indicate the colocalization of PAK5 with Cdc42 or Integrin β1, β3. Scale bars represent 10 μm. All experiments were performed three times

### 3.4 PAK5 interacting with Cdc42 and Integrin β1, β3 accelerated CRC cells migration and invasion

To further investigate whether Cdc42 and Integrins are indispensable for PAK5‐promoted cell migration and invasion, and to assess whether the kinase activity of PAK5 is also required for such process, we constructed a vector containing the full‐length wild‐type PAK5, and vectors containing one of three dominant‐negative PAK5 mutants: PAK5 (K478M) harbors a single‐point mutation within the kinase domain rendering its inactive kinase activity^13^, ^33^; PAK5△CRIB lacks the CRIB region so it cannot bind with Cdc42^13^; and PAK5△IBD lacks the Integrin‐binding domain (IBD),^32^ resulting in deficient ability to interact with Integrins (Figure 5A). Vectors construction was confirmed by western blotting (Figure 5B). The binding capability of PAK5 with Cdc42 or Integrin β1, β3 was verified by co‐IP (Figure 5C,D) assays, indicating that the CRIB and IBD regions are indispensable for PAK5 to directly interact with Cdc42 and Integrin β1, β3 in HCT116 cells.

**Figure 5:** PAK5 interacting with Cdc42 and Integrin β1, β3 accelerated CRC cells migration and invasion. A, Schematic representing generated flag‐tagged PAK5 constructs, including wild‐type PAK5, and three dominant‐negative PAK5 mutants: PAK5 (K478M), PAK5△CRIB, and PAK5△IBD. B, Protein expression of wild‐type or mutant PAK5 plasmids in HCT116 cells were determined by western blots. C, The interaction of PAK5△CRIB with CDC42 was detected by co‐IP assays in HCT116 cells. D, The interaction of PAK5△IBD with Integrin β1, β3 was detected by co‐IP assays in HCT116 cells. E, HCT116 cell proliferation was determined by CCK‐8 assays after transfection with wild‐type or mutant PAK5 plasmids. Absorbances were recorded every day for 7 d. F, HCT116 cells colony formation ability were assessed after transient transfection with wild‐type or mutant PAK5 plasmids for 7 d. Colony number for each group was counted and analyzed. G, HCT116 cells were transfected with wild‐type or mutant PAK5 plasmids. Cell lysates were examined by western blots to determine the protein levels of p‐CRAF (Ser338), p‐BAD (Ser112), p‐BAD (Ser136), and BAD. α‐tubulin was used as the internal control. D, HCT116 cells migration and invasion after transient transfection with wild‐type or mutant PAK5 plasmids were detected by transwell assays. The quantitative data were presented as means ± *SD* from three independent experiments. ^***^ *P* < .001

We next questioned whether the kinase activity and the participation of Cdc42 and Integrin β1, β3 are essential for PAK5‐promoted CRC cells proliferation, migration, and invasion. HCT116 cells transiently transfected with either empty vector or vectors containing wild‐type or mutant PAK5 showed a markedly accelerated cell growth after transfecting wild‐type PAK5, PAK5△CRIB, or PAK5△IBD, but not empty vector or PAK5 (K478M) (Figure 5E), indicating that the kinase activity is essential for PAK5‐induced cell proliferation in HCT116 cells, which was validated by the colony‐forming assay (Figure 5F). To further investigate the mechanism of PAK5‐accelerated CRC cells proliferation, the expression of proapoptotic protein BAD was assessed. Consistent with previous studies, PAK5 transfection elevated the phosphorylation level of BAD on serine 112 and 136. On the contrary, kinase‐inactive PAK5 rendered downregulated phosphorylation of CRAF (a downstream substrate of PAK5)^34^ on serine 338 and decreased BAD phosphorylation levels (Figure 5G), indicating that BAD phosphorylation was involved in PAK5‐promoted CRC cell proliferation. By contrast, transwell experiments showed that cell migration and invasion abilities were restrained after transfecting PAK5△CRIB or PAK5△IBD, but not in cells treated with wild‐type PAK5 or PAK5 (K478M) (Figure 5H), demonstrating that Cdc42 and Integrin β1, β3 are involved in PAK5‐accelerated CRC cells migration and invasion.

The article "PAK5 facilitates the proliferation, invasion and migration in colorectal cancer cells" was retracted in 2024. Reasons: duplicated images; duplicated data; overlap with earlier publications; original data or images not available.

### 3.5 PAK5 facilitated CRC cells proliferation and metastasis in xenograft model

To further validate the functional role of PAK5 in CRC cells proliferation and metastasis in vivo, lentivirus encoding either empty vector or PAK5 *shRNA* was employed to transduce HCT116 cells, designated as pLKO.1_*Ctrl* and pLKO.1_*shPAK5*. Nude mice were orthotopically implanted with cells either expressing pLKO.1_*Ctrl* or pLKO.1_*shPAK5*. Five mice were allocated for each group, and we observed a significantly reduced tumor volume in pLKO.1_*shPAK5* group as compared with pLKO.1_*Ctrl* group (Figure 6A). The metastatic nodules on the liver were also monitored and recorded, showing diminished metastatic tumor nodules number in pLKO.1_*shPAK5* group vs pLKO.1_*Ctrl* group (Figure 6C), demonstrating that PAK5 accelerated the proliferation and metastasis of CRC cells in vivo. Furthermore, hematoxylin and eosin (H&E) staining analysis revealed less hypercellular and alleviative nuclear polymorphism in pLKO.1_*shPAK5* group as compared with pLKO.1_*Ctrl* group. In addition, decreased numbers of Ki67‐positive proliferating cells were discovered in pLKO.1_*shPAK5* group *vs* pLKO.1_*Ctrl* group (Figure 6E), confirming that PAK5 promoted CRC cells proliferation and metastasis in vivo. In contrast, SW480 cells transduced with lentivirus packing either empty vector or PAK5 were named as pLenti_*mock* or pLenti_*PAK5*. Nude mice orthotopically injected with pLenti_*PAK5* showed remarkably enhanced tumor volume and increased numbers of metastatic nodules on the liver as compared with pLenti_*mock* group (Figure 6B,D). Similarly, we observed more severe morphological changes and more Ki‐67‐positive cells in pLenti_*PAK5* group *vs* pLenti_*mock* group (Figure 6F), validating that CRC cells proliferation and metastasis were facilitated by PAK5 in xenograft models.

**Figure 6:** PAK5 facilitated CRC cells proliferation and metastasis in xenograft model. A, C, E Nude mice (n = 5 for each group) were orthotopically transplanted with HCT116 cells stably expressing pLKO.1_*Ctrl* or pLKO.1_*shPAK5*. A, Tumor growth in each group was measured and recorded for 25 d. Excised tumors in different groups were shown. C, Numbers of liver metastasis nodules from each mouse were counted. Representative photographs were shown. E, Tumor sections were stained with either H&E or Ki‐67 antibody. Representative photographs were shown. Scale bars for H&E staining represent 100 μm; Scale bars for Ki67 staining represent 50 μm. B, D, F, Nude mice (n = 5 for each group) were orthotopically transplanted with SW480 cells stably expressing pLenti_*mock* or pLenti_*PAK5*. B, Tumor growth in each group was measured and recorded for 25 d. Excised tumors in different groups were shown. D, Numbers of liver metastasis nodules from each mouse were counted. Representative photographs were shown. F, Tumor sections were stained with either H&E or Ki‐67 antibody. Representative photographs were shown. Scale bars for H&E staining represent 100 μm; Scale bars for Ki67 staining represent 50 μm. Data were presented as means ± *SD*, ^*^ *P* < .05; ^**^ *P* < .01; ^***^ *P* < .001

## 4 DISCUSSION

Since the first PAK family member, PAK1 was characterized by Manser et al in 1994,^35^ abundant studies have pointed out the involvement of PAKs in a variety of cellular activities, including cytoskeletal remodeling, cell survival, and embryonic development.^29^, ^36^, ^37^ Recently, accumulating evidences demonstrated a key role of PAKs in tumorigenesis.^9^, ^38^, ^39^ Despite an enhanced PAK function in various human tumors, which is positively correlated with advanced tumor stages and poor prognosis, PAK isoforms are not frequently mutated. Instead, it's overexpression or hyperactivation by mutations in the upstream modulators such as RAC or Cdc42 that enables them to initiate and promote carcinogenesis.^30^ As the final identified PAK member, PAK5 was proved to be linked with tumor progression. High PAK5 expression was found in multiple types of cancer such as pancreatic and hepatic cancers,^14^, ^40^ whereas its role in colorectal cancer is still not fully understood. In this study, we verified an increased expression of PAK5 in primary CRC specimens as well as in human colon cancer cells. Importantly, statistical analysis of TNM stages supported a positive relevance between high PAK5 expression and advanced CRC malignancy, pointing out a potential of PAK5 to serve as a prognostic biomarker in CRC in the future.

The article "PAK5 facilitates the proliferation, invasion and migration in colorectal cancer cells" was retracted in 2024. Reasons: duplicated images; duplicated data; overlap with earlier publications; original data or images not available.

The balance between proliferation and apoptosis is vital to cell survival. Several PAK isoforms have been shown to exert the effects of antiapoptosis and promoting cell proliferation, which is pivotal in tumorigenesis. PAK5 has been revealed to accelerate cell growth via restriction of apoptosis in several cell types. It is said that such antiapoptotic effects are mediated through CRAF, a known substrate of PAK5.^34^, ^41^ CRAF phosphorylated by PAK5 at Ser338 drives its translocation to the mitochondria, subsequently binding to and phosphorylating BAD. BAD phosphorylation stops it from interacting with BCL‐2, thus resulting in promoting cell proliferation.^34^, ^42^ Our in vitro and in vivo studies demonstrated a facilitation of PAK5 in CRC cell growth. We further revealed that ectopic expression of PAK5 alleviated 5‐FU‐induced apoptosis. Similarly, Zhang *et al* reported that PAK5 overexpression remarkably decelerated cisplatin‐stimulated apoptosis in hepatocellular carcinoma cells.^43^ In addition, our results uncovered that a functional kinase activity is essential for PAK5‐promoted cell growth, which was validated by the dominant‐negative PAK5 mutants PAK5 (K478M). However, it still remains to be elucidated whether all PAK members promote cell survival in a kinase‐dependent mechanism, as PAK4 has been shown to prevent apoptosis through both kinase dependent and independent manner.^44^, ^45^, ^46^

Apart from its key role in apoptosis, PAK5 is also known to be involved in cell migration and invasion, which might trigger metastatic tumor cells to spread to distant organs.^47^ Cell migration and invasion are complex process, involving extensive cytoskeleton remodeling, perturbation of cell adhesion, and digestion of extracellular matrix to offer extra space for cell movement.^48^, ^49^ As the key upstream regulator of PAK5, the small GTPase CDC42 is known to participate in the modulation of cell motility via promoting the formation of membrane protrusions such as filopodia and lamellipodia.^28^, ^50^ Cdc42 deficiency led to a defect in global cell‐matrix interactions in mouse embryonic fibroblasts (MEFs), which could not be rescued by reintroducing mutants of Cdc42 that lack PAK binding activity.^51^ Similarly, Integrins, a family of transmembrane glycoproteins, play a major role in invasive and metastatic processes.^28^ Overexpression of Integrins is often correlated with invasive cancers with a poor prognosis.^52^ Emerging evidence further pointed out that Integrins as crucial effectors are involved for PAK controlled cell motility.^31^ However, it still remains controversial whether Cdc42 and Integrins are indispensable in PAKs‐modulated cell adhesion and migration, as a Cdc42‐independent mechanism in PAK4‐derived cell adhesion turnover in breast cancer cells has been reported.^53^ Instead of Cdc42, the nonconventional Rho GTPase, RhoU is stabilized by binding with PAK4, thereby associated with cell adhesion turnover and migration. In our current study, in vitro and in vivo results revealed a promoting function of PAK5 in CRC cells migration and invasion. We further showed that the participation of Cdc42 and Integrin β1, β3 is necessary for PAK5‐driven cell mobility in CRC. Interestingly, we found that the kinase activity was not essential for PAK5‐accelerated cell migration and invasion. Whether the kinase activity is pivotal in PAKs‐stimulated cell motility remains to be fully characterized, as both kinase‐dependent and ‐independent mechanisms have been reported.^54^ Our study reminisces a previous evidence showing that both kinase‐dead or constitutively‐active PAK1 could induce dramatic actin organization.^55^ Moreover, our results suggested that PAK5‐targeting cancer therapeutics might be designed to inhibit the total PAK5 level, rather than solely blocking the catalytic activity.

The article "PAK5 facilitates the proliferation, invasion and migration in colorectal cancer cells" was retracted in 2024. Reasons: duplicated images; duplicated data; overlap with earlier publications; original data or images not available.

In summary, we herein presented a new view regarding the function of PAK5 in CRC tumorigenesis. Our study validated that PAK5 was remarkably correlated with CRC malignant progression. Moreover, in vitro and in vivo findings demonstrated that PAK5 could serve as a novel therapeutic target in restraining CRC proliferation and metastasis. The uncovered mechanisms will deepen the comprehension about the mechanisms of CRC progression, as well as providing new insights for therapeutic intervention in colorectal cancer.

## CONFLICT OF INTERESTS

The authors declare that they have no competing interests.

## AUTHORS’ CONTRIBUTIONS

SLH, YZ, and CFW performed experiments; WG designed the study; WG and WH managed the project; All authors contributed intellectually to the project through discussion, analyzed the results, and critically reviewed the manuscript.

## CONSENT FOR PUBLICATION

Informed consent was obtained from all patients and their relatives.

## ETHICS APPROVAL AND CONSENT TO PARTICIPATE

This study was approved by the Ethic Committee of Southern Medical University.

## Supporting information

Table S1

## Data Availability

The data used to support the findings of this study are available from the corresponding author upon request.
